# Giant Traumatic Diaphragmatic Hernia: A Report of Delayed Presentation

This article has been retracted.

**DOI:** 10.7759/cureus.20315

**Published:** 2021-12-10

**Authors:** Abbas H Alsuwayj, Ali H Al Nasser, Abdulaziz M Al Dehailan, Abdullah Z Alburayman, Khalid A Alhuwaiji, Khurayzan F Binsifran, Ibrahim M Almulhim, Abdullah F Almulhim, Mohammed A Al Amer, Mohannad A Almulhim, Abdullatif Y Almulhim, Abdullah A Almulhim, Insaf A Alhazoom, Ahmed A Albakheet, Faisal Al-Hawaj

**Affiliations:** 1 College of Medicine, King Faisal University, Al-Ahsa, SAU; 2 College of Medicine, Imam Abdulrahman Bin Faisal University, Dammam, SAU

**Keywords:** case report, computed tomography, respiratory distress, diaphragm, hernia, trauma

## Abstract

Diaphragmatic rupture is an uncommon injury after blunt abdominal trauma. The diaphragmatic defect may not be obvious in imaging studies immediately after the initial injury. Patients may have delayed presentation when the diaphragmatic defect enlarges and allows abdominal content to herniate into the thoracic cavity. Here, we present the case of a 30-year-old man who presented with the emergency department complaining of shortness of breath at rest for two days duration. He reported having shortness of breath for the last five years, but he attributed it to his smoking. The shortness of breath was associated with cough productive and vague abdominal pain. The patient had an unremarkable relevant medical history. He reported having a motor vehicle accident five years ago that was severe but he did not sustain any significant injuries or fractures. Upon examination, the patient appeared in respiratory distress. Respiratory examination revealed diminished air entry on the left hemithorax and the abdominal examination revealed increased generalized tenderness with increased bowel sounds. The patient underwent a thoracic computed tomography scan, which unexpectedly demonstrated a huge left-sided diaphragmatic defect with bowel loops observed to occupy the left hemithorax completely. The patient was stabilized and shifted to emergency laparotomy during which the hernia content was reduced and the defect was closed with a mesh. The patient reported the resolution of his symptoms after the surgery. Intensive chest physiotherapy exercises were performed. After six months of follow-up, the patient remained asymptomatic with no active complaints. The diaphragmatic hernia may have delayed presentations after several years of blunt abdominal trauma. The case highlighted the importance of initial imaging studies after blunt trauma may not identify the diaphragmatic defect.

## Introduction

Diaphragmatic rupture is a relatively rare and serious injury that accounts for less than 1% of all traumatic injuries [1]. Such incidences are continuously rising because of the increased number of motor vehicle accidents; however, improved trauma care has led to better diagnosis and treatment regimens [2]. In over one-third of cases, the mechanism of traumatic diaphragmatic injury includes blunt abdominal trauma, which can be due to motor vehicle accidents in over 90% of cases [3]. Such injuries cause a significant increase in the intra-abdominal pressure resulting in traumatic rupture of the diaphragm. While diaphragmatic rupture can be obvious on chest radiograph, the injury can be difficult to diagnose in certain cases [2]. In addition to herniation, diaphragmatic rupture can result in associated injuries, including diaphragmatic paralysis and pulmonary contusion [3]. Patients may have no symptoms initially after the diaphragmatic injury, but the defect may enlarge with time and result in large herniation of the abdominal organs [1]. Hence, it is crucial to keep a high index of suspicion for diaphragmatic injuries in patients who sustained significant blunt abdominal trauma. Here, we present the case of a middle-aged man with a delayed presentation of a giant diaphragmatic hernia.

## Case presentation

We present the case of a 30-year-old man who came to the emergency department complaining of shortness of breath at rest for two days duration. He reported that he had been experiencing shortness of breath over the last five years and he believed that it could be because of his heavy smoking habits so he did not seek medical care. However, for the last one month, the shortness of breath progressed to the degree that interfered with his activities of daily living. He reported that the difficulty in breathing is aggravated by lying flat on the bed. This caused him to have poor sleep quality and morning headaches. The shortness of breath was associated with cough productive of yellowish sputum with no hemoptysis. The patient reported no history of calf swelling, wheezing, fever, or weight loss. However, the patient reported that he experienced vague abdominal pain and early satiety. This was associated with decreased bowel motion.

Besides thalassemia minor, the patient had an unremarkable history of comorbid conditions. However, the patient reported that he had a motor vehicle accident five years ago. The accident was severe, but he did not sustain any significant injuries or fractures. He did not undergo any surgical operations. He did not take any medications apart from multivitamins. There was no history of food or drug allergy. He was a heavy smoker (30 pack-years) and consumed alcohol on a few occasions. The family history was remarkable for coronary artery disease.

Upon examination, the patient appeared in respiratory distress. He was not able to complete a full sentence. His vital signs revealed tachycardia (130 bpm [breaths per minute]) and tachypnea (25 bpm). However, his temperature (37.1°C) and blood pressure (129/80 mmHg). The oxygen saturation was 96% in room air. Respiratory examination revealed diminished air entry to the left hemithorax. Cardiac examination revealed normal S1 and S2 with no added sounds or murmurs. However, the apex beat was not palpable. Abdominal examination revealed increased generalized tenderness with increased bowel sounds. The initial laboratory investigation, including hematological and biochemical parameters, did not reveal any abnormalities (Table 1).

**Table 1:** Summary of the results of laboratory findings

Laboratory Investigation	Unit	Result	Reference Range
Hemoglobin	g/dL	14.5	13.0–18.0
White Blood Cell	1000/mL	8.2	4.0–11.0
Platelet	1000/mL	374	140–450
Erythrocyte Sedimentation Rate	mm/hr	15	0–20
C-Reactive Protein	mg/dL	3.8	0.3–10.0
Total Bilirubin	mg/dL	0.5	0.2–1.2
Albumin	g/dL	3.7	3.4–5.0
Alkaline Phosphatase	U/L	55	46–116
Gamma-glutamyltransferase	U/L	21	15–85
Alanine Transferase	U/L	16	14–63
Aspartate Transferase	U/L	20	15–37
Blood Urea Nitrogen	mg/dL	10	7–18
Creatinine	mg/dL	0.8	0.7–1.3
Sodium	mEq/L	138	136–145
Potassium	mEq/L	3.8	3.5–5.1
Chloride	mEq/L	106	98–107

In view of the severe symptoms and the physical examination findings, the patient underwent a thoracic computed tomography scan. Unexpectedly, the scan demonstrated a huge left-sided diaphragmatic defect with bowel loops were observed to occupy the left hemithorax completely. The hernia was exerting a pressure effect resulting in mediastinal shift (Figure 1). The thoracic and gastrointestinal surgery teams were immediately informed about these findings.

**Figure 1:** CT images of the thorax and upper abdomen CT: Computed Tomography Coronal (A) and sagittal (B) CT images demonstrate a diaphragmatic defect (encircled) resulting in a massive herniation of the abdominal content, including the small intestine (yellow arrow) and the spleen (blue arrow)

The patient was stabilized and shifted to emergency laparotomy. During diagnostic exploration, the diaphragm was found to have a tear, measuring 16 cm × 13 cm, with herniation of the omentum, intestinal loops, and the spleen. The content of the hernia was reduced and the defect was closed with a non-absorbable mesh. The incisions were closed. A left thoracotomy tube was placed. The patient had an uneventful recovery. The patient reported the resolution of his symptoms after the surgery. Intensive chest physiotherapy exercises were performed. The patient was discharged one week postoperatively. He was given several physiotherapy sessions. After six months of follow-up, the patient remained asymptomatic with no active complaints.

## Discussion

We present the case of a diaphragmatic hernia that presented five years after the initial trauma. Delayed presentation of diaphragmatic rupture is usually due to thoracic herniation of the abdominal content. It is estimated that up to 30% of diaphragmatic hernias have delayed presentations [4]. There are several hypotheses that were suggested to provide an explanation of the delayed presentation of diaphragmatic hernias. First, the diaphragmatic rupture may not necessarily occur immediately after the injury and may develop later in the necrotic diaphragmatic muscle. Second, the diaphragmatic rupture may be passed unnoticed if it was not initially associated with hernia [5].

The duration between the injury and the presentation is variable. The available literature showed that the duration of a hernia might range from one day to 50 years [6]. In the present case, it seemed that the reason behind the late presentation after five years is due to the patient attributing his symptoms to his smoking behavior and not seeking medical care earlier. The clinical presentation of delayed diaphragmatic hernia is non-specific. It may present with shortness of breath, abdominal pain, chest pain, and cough [7]. In our case, the patient initially developed longstanding shortness of breath that he ignored, then he presented with respiratory distress. Some case reports included presentations with intestinal obstruction, melena, hematemesis, and hemodynamic instability.

Regarding the site of the hernia, it is believed that right-sided hernias are less common because of the protective effect on the liver. Further, up to 90% of case reports of delayed diaphragmatic hernias had left-sided defects [5]. However, postmortem studies showed an equal prevalence of the right and left diaphragmatic defects. This suggests that patients with right-sided hernias have higher pre-hospital mortality. Bilateral hernias are very rare but have been reported [6].

Regarding the investigation modalities to diagnose a diaphragmatic hernia, it should be noted that more than 50% of diaphragmatic ruptures are not detected by chest radiographs. A computed tomography scan has higher sensitivity and may detect up to 70% of diaphragmatic ruptures. Meticulous inspection during diagnostic laparoscopy should be performed if there is any suspicion in patients with trauma [6]. The management of diaphragmatic hernia involves reduction of the herniated content, repairing the defect, and pleural drainage [4]. The prognosis of a diaphragmatic hernia depends on the presence of strangulated bowel. The mortality is low in uncomplicated cases. However, it may reach more than 80% in the setting ischemic bowel [5].

## Conclusions

The diaphragmatic hernia may have delayed presentations after several years of blunt abdominal trauma. The initial imaging studies after blunt trauma may not identify the diaphragmatic defect. The case highlighted the importance of considering diaphragmatic rupture in the differential diagnosis of respiratory symptoms in patients with a previous history of significant blunt abdominal trauma. Surgical repair of the hernia is the mainstay in the treatment and it can be done by laparotomy or thoracotomy.
